# *In Vivo* Reconstruction of the Acetabular Bone Defect by the Individualized Three-Dimensional Printed Porous Augment in a Swine Model

**DOI:** 10.1155/2020/4542302

**Published:** 2020-11-30

**Authors:** Jun Fu, Yi Xiang, Ming Ni, Xiaojuan Qu, Yonggang Zhou, Libo Hao, Guoqiang Zhang, Jiying Chen

**Affiliations:** ^1^Department of Orthopaedics, The First Medical Centre, Chinese PLA General Hospital, Beijing 100853, China; ^2^Department of Orthopaedics, The Logistics Support Forces of Chinese PLA 985 Hospital, Taiyuan, Shanxi 030001, China; ^3^Otolaryngological Department, The Logistics Support Forces of Chinese PLA 985 Hospital, Taiyuan, Shanxi 030001, China

## Abstract

**Methods:**

As an acetabular bone defect model created in Bama miniswine, an augment individually fabricated by 3D print technique with Ti6Al4V powders was implanted to repair the defect. Nine swine were divided into three groups, including the immediate biomechanics group, 12-week biomechanics group, and 12-week histological group. The inner structural parameters of the 3D printed porous augment were measured by scanning electron microscopy (SEM), including porosity, pore size, and trabecular diameter. The matching degree between the postoperative augment and the designed augment was assessed by CT scanning and 3D reconstruction. In addition, biomechanical properties, such as stiffness, compressive strength, and the elastic modulus of the 3D printed porous augment, were measured by means of a mechanical testing machine. Moreover, bone ingrowth and implant osseointegration were histomorphometrically assessed.

**Results:**

In terms of the inner structural parameters of the 3D printed porous augment, the porosity was 55.48 ± 0.61%, pore size 319.23 ± 25.05 *μ*m, and trabecular diameter 240.10 ± 23.50 *μ*m. Biomechanically, the stiffness was 21464.60 ± 1091.69 N/mm, compressive strength 231.10 ± 11.77 MPa, and elastic modulus 5.35 ± 0.23 GPa, respectively. Furthermore, the matching extent between the postoperative augment and the designed one was up to 91.40 ± 2.83%. Besides, the maximal shear strength of the 3D printed augment was 929.46 ± 295.99 N immediately after implantation, whereas the strength was 1521.93 ± 98.38 N 12 weeks after surgery (*p* = 0.0302). The bone mineral apposition rate (*μ*m per day) 12 weeks post operation was 3.77 ± 0.93 *μ*m/d. The percentage bone volume of new bone was 22.30 ± 4.51% 12 weeks after surgery.

**Conclusion:**

The 3D printed porous Ti6Al4V augment designed in this study was well biocompatible with bone tissue, possessed proper biomechanical features, and was anatomically well matched with the defect bone. Therefore, the 3D printed porous Ti6Al4V augment possesses great potential as an alternative for individualized treatment of severe acetabular bone defects.

## 1. Introduction

Total hip arthroplasty (THA) represents one of the most successful surgeries in the 20^th^ century and has been employed for releasing pain, correcting the deformity, and improving the function of the hip joint [1, 2]. The management of severe acetabular bone defects in primary or revision THA remains a challenge for surgeons, and the ideal defect reconstruction is a critical factor for a successful THA [3]. Traditionally, major acetabular defects in primary and revision THA have been reconstructed by impaction bone grafting (IBG), metal augments, and cup/cage constructs [2]. Recently, given the improved biocompatibility and biomechanical properties of the trabecular metal (TM), TM augments and cups are most commonly used and have achieved good clinical midterm outcomes in patients. Since TM augments are mass-produced with a unitary shape, they tend to anatomically mismatch with acetabular bone defects, and reaming the residual bone stock of acetabular defects is required in most cases [4–6]. Therefore, individualized augments are needed in these cases to better reconstruct the acetabular bone defects.

Titanium and titanium alloy are widely used to fabricate orthopaedic prostheses and instruments for their good biocompatibility, high strength, and low corrosion rates [7]. Multiple studies have been conducted to optimize the microstructure of the Ti6Al4V alloy, and porous Ti6Al4V alloy implants mechanically compatible with the cancellous bone have been developed [8, 9]. Studies showed that the pore size between 200 *μ*m and 500 *μ*m and a porosity of 50-75% were optimal for bone ingrowth and osteointegration [10, 11]. Further studies examined their biocompatibility and biomechanical features of the alloy *in vitro*, *in vivo*, and in clinical patients [12–14].

With the rapid development of the 3D printing technology, the 3D printed medical models, with an advantage of personalized treatment, are being extensively used in orthopaedic prostheses [15, 16]. Although a case report described the clinical application of the 3D printed augments in the repair of the acetabular defect [15], implant-bone integration has not been well assessed. In a previous study, we established a finite element analysis (FEA) model of the acetabular bone defect, which was reconstructed by 3D printed porous Ti6Al4V augments, and evaluated the stress distribution and clinical safety of augments, screws, and bones [17]. Until now, the performance of these 3D printed porous augments in animal models has not been systemically elucidated.

In this study, we established a miniswine model of the acetabular bone defect and implanted the 3D printed porous augments that were anatomically compatible with the bone defect. We further evaluated the bone ingrowth, biomechanics, and matching degree of the 3D printed porous augments in the animals.

## 2. Materials and Methods

### 2.1. Establishment and Validation of the Animal Model of the Acetabular Bone Defect

All animal experiments in this study were approved by the Experimental Animal Ethics Committee of the General Hospital of Chinese People's Liberation Army, Beijing, China. Bama miniswine (female, 14-18 months old with a body weight of 25-30 kg) were used to establish and validate the animal model of the acetabular bone defect. The swine were routinely maintained in the Experimental Animal Center of the General Hospital of Chinese People's Liberation Army. These miniswine were divided into three groups, with three animals in each group. Animals in group 1 were subjected to the biomechanical test immediately after augment implantation; swine in group 2 were biomechanically tested 12 weeks after augment implantation; pigs in group 3 were histologically examined 12 weeks after augment implantation. The miniswine were kept and fed in separate cages according to standard animal care protocols [18]. All the surgeries were performed on the right acetabulum of the miniswine. The anesthetic methods included intramuscular and general anesthesia. Intramuscular anesthetics were a mixture of ketamine hydrochloride and xylazine hydrochloride (1 : 1 ratio, 15-25 mg/kg). The general anesthetic was 3% pentobarbital sodium (30 mg/kg). The vital signs (heart rate, breathing, and oxygen saturation) of the miniswine were carefully monitored, and intravenous fluid therapy involving glucose and lactated Ringer's solution was used during the operation.

At the first surgical phase of defect model establishment (Figures 1(a)–1(d)), the operation sites were removed of hair, shaved, disinfected, and draped. A straight 10 cm skin incision was made at the hip via the anterolateral approach. Then, the anterosuperior wall of the acetabulum was exposed clearly and a Paprosky IIB acetabular bone defect (an equilateral triangle with sides of about 2 cm) was made as previously reported [19]. The wound site was sutured for closure, and the acetabular bone defect was left untreated for approximately 1 week (waiting for fabrication by the 3D printed Ti6Al4V augment).

### 2.2. Design and Fabrication of the 3D Printed Porous Ti6Al4V Augment

Computed tomography (CT) scan of the animal pelvis was taken immediately after the establishment of the bone defect model. The pelvis and porous Ti6Al4V augment were three-dimensionally reconstructed on a direct metal laser sintering (DMLS) system (EOSINT M280, Germany) using a computer-aided design (CAD) software package (Mimics Research 20.0, Materialise, Belgium). A medical Ti6Al4V powder (EOS, Germany) with particles sized from 15 *μ*m to 53 *μ*m was used. The porous augments were 3D printed at a scanning rate of 7 m/s and a power of 200 W.

The inner pore parameters were as follows: a cubic-shaped lattice structure had a pore size of 400 *μ*m, a strut size of 200 *μ*m, and a porosity of 60%. The thickness of the porous Ti6Al4V coating was 1 mm, while the rest of the augment was of solid Ti6Al4V. Meanwhile, the position, direction, length, and diameter of screws and Kirschner wires (for temporary intraoperative fixation of the augment) were designed according to the residual bone stock of acetabular defects. The length of the screw ranged between 16 mm and 20 mm. The diameters of screws and K-wires were 4.0 mm and 1.5 mm, respectively. After printing, the 3D printed porous augments were cleaned, polished, sterilized, and then implanted. (Figures 2(a)–2(d) and 2(f)).

### 2.3. Porosity and Mechanical Evaluation of the 3D Printed Porous Augments

Printed specimens, with a diameter of 10 mm and a height of 20 mm, were used for evaluation of porosity and mechanical properties against the International Organization for Standardization (ISO 13314:2011). The total porosity and open porosity were measured using the gravimetric method and Archimedes' principle, respectively. The pore morphology, including pore size and strut size, was evaluated by using scanning electron microscopy (SEM, Zeiss Supra 55, Germany). The compressive strength of the porous Ti6Al4V augment was determined by employing a computer-controlled mechanical testing machine (Instron-8874, Instron, USA) at a loading speed of 1 mm/min. The elastic modulus of the porous Ti6Al4V augment was calculated on the linear region of the stress-strain curve. The final measurements were averaged from five specimens in every group.

### 2.4. Implantation of the 3D Printed Porous Ti6Al4V Augment

At the second surgical phase of the 3D printed porous Ti6Al4V augment implantation (Figures 1(e) and 1(f)), preoperative preparation and exposure were similar to the first phase. The individual porous augment was placed on the acetabular defect surface, and two 1.5 mm K-wires were used for temporary fixation. The augment matched well with the defect in terms of shape and size as observed by the naked eye. Then, two screws of appropriate length were inserted into the augment screw holes. Immediate stability of the augment was confirmed by shaking tests. The muscle tissues and skin were sutured layer by layer. After surgery, two injections of penicillin G (at 80 wu/time) were administered 48 hours after the implantation and at incision dressing.

All miniswine were subjected to pelvis CT scan immediately after surgery, and the DICOM data were used for the three-dimensional reconstruction of the augment. Then, the matching degree was calculated in terms of the overlapping ratio between the designed augment and the implanted one (Figures 3(a)–3(d)).

### 2.5. Microcomputed Tomography

To evaluate the ingrowth of the bone tissues around the porous Ti6Al4V augment, specimens, prior to histological examination, were observed under micro-CT (SkyScan 1172, Belgium) under the following conditions: 100 kV acceleration voltage at 75 *μ*A (current). All specimens were scanned at a complete 360° rotation, with an exposure time of 1600 ms and a resolution of 13.75 *μ*m.

### 2.6. Biomechanical Test (Push-Out Test)

The push-out test was conducted on a computer-controlled mechanical testing machine (Instron-E3000, Instron, USA) at a loading speed of 0.5 mm/min. The augment-containing bone specimen with an intact iliac wing from a sacrificed miniswine was embedded into a sensor, and the other side was a metal cone serving as the femoral head. The ultimate shear strength was recorded when the implanted augment started to move after continuous loading. The structure of the mechanical testing platform is shown in Figure 4(a).

### 2.7. Histological and Histomorphometric Analyses

Three miniswine (group 3) were prepared for histological analysis. To evaluate the bone ingrowth distance over time, fluorochrome (two injections), tetracycline (25 mg/kg) and calcein green (at 25 mg/kg), were administered intramuscularly 14 and 13 days (tetracycline) and 4 and 3 days (calcein green) before sacrificing at 12 weeks after surgery.

Augment-containing bone specimens were then fixed in formalin, dehydrated, and then embedded. Next, they were sectioned with a low-speed cutter (IsoMet™, Buehler, USA) in serial sections of 300 *μ*m and ground to a thickness of 50 *μ*m. The newly formed bone was determined by the distance between the two fluorochrome labels using an epifluorescent microscope (DMi8, Leica, Germany) (Figure 5(a)). The amount of new bone and bone ingrowth to the porous Ti6Al4V coating was calculated, by using an image processing software package (Image-Pro Plus 6.0, Media Cybernetics, USA), as a percentage of the total bone-implant interface area (Figure 5(b)). The bone mineral apposition rate (MAR) was calculated by dividing the distance between the two fluorochrome labels by 10 days (the time interval between the two injections of fluorochrome) and expressed as mm per day. Tb/T referred to the ratio of the tissue bone area to the total view area of the region of interest, which included the new bone area and material area.

### 2.8. Statistical Analysis

All the analyses were performed using SPSS for Windows (version 18.0, SPSS Inc., Chicago, Illinois, USA). Comparison of rates was made by the chi-squared test, while numerical data were compared by using a paired sample *t*-test (normal distribution and homoscedasticity) or a Wilcoxon rank test. A *p* value less than 0.05 was considered statistically significant.

## 3. Results

### 3.1. Porosity and Mechanical Characterization

Measurement of porosity on the 3D printed porous Ti6Al4V augments by using the gravimetric method and against Archimedes' principle revealed that total porosity and open porosity of the samples were 55.48 ± 0.61% and 49.02 ± 2.22%, respectively. The pore size and strut size measured by using SEM were 319.23 ± 25.05 *μ*m and 240.10 ± 23.50 *μ*m, respectively. Biomechanically, the stiffness of porous augment was 21464.60 ± 1091.69 N/mm, compressive strength was 231.10 ± 11.77 MPa, and elastic modulus was 5.35 ± 0.23 GPa, respectively.

### 3.2. Experimental and Photographic Results

We achieved a 100% success rate with the establishment of the acetabular bone defect, as evidenced by successful implantation, no loosening and displacement, and good joint activity in all the animals. However, the failure rate of the 3D printed augment implantation was 18.18% (2 of 11 swine). One swine developed a deep infection after implantation, and the other one had screw loosening and augment detachment from the acetabular bone.

Micro-CT imaging was used to assess the bone ingrowth around the porous augment. As shown in Figure 2(e), bone formation occurred within porous augments. The three-dimensional reconstruction of CT data showed that the individual augment anatomically matched well with the defect, and the degree of matching in these 9 swine was 91.40 ± 3.01% (Figure 3(e)).

### 3.3. Push-Out Test Results

Shear strength reflects prosthetic stability after implantation and was detected by push-out tests. The ultimate shear strength immediately and 12 weeks after surgery was 929.46 ± 295.99 N and 1521.93 ± 98.38 N, respectively (*p* = 0.0302) (Figure 4(b)). Since, in the actual situation, the augment and the screws were also under the compressive stress, the shear strength measured in this biomechanical model might be representative of the ultimate shear strength after surgery.

### 3.4. Histological and Histomorphometric Evaluation of Bone Formation

Tetracycline and calcein green bands are indicative of new bone formation and allow the measurement of the mineral apposition rate during the observation period. The bone mineral apposition rate (*μ*m per day) 12 weeks post operation was 3.77 ± 0.93 *μ*m/d (Figure 5(c)). The percentage bone volume of new bone 12 weeks after surgery was 22.30 ± 4.51% (Figure 5(d)).

## 4. Discussion

To better repair severe acetabular bone defects, the present work characterized the performance of the 3D printed porous Ti6Al4V augments in an animal model. The results in miniswine demonstrated that the augments fabricated in our study had good bone tissue biocompatibility and biomechanical properties. The postoperative CT data showed that the 3D printed augments morphologically well matched with the bone defect and the acetabular components.

The effects of porosity, pore size, and shape on the biological behaviors of porous Ti6Al4V prostheses have been previously investigated [20–23]. Heinl et al. demonstrated that the three-dimensional structures with an interconnected mean porosity of 61.3% and a pore size of 450 *μ*m were suitable for tissue ingrowth and vascularization [20]. The 3D printed porous Ti6Al4V scaffold with a total porosity of 58% and a pore size of 500 ± 50 *μ*m possessed mechanical properties similar to human bone and promoted osseointegration and tissue integration in animal experiments [21]. Wieding and Wolf measured the uniaxial compression, bending, and torsion strength of the porous Ti6Al4V scaffold and exhibited that pore size of 400 *μ*m was numerically optimal for porous bone scaffold structures to match the elastic properties of human bone [22]. They also showed that the cubic design had the lowest elastic modulus and the fastest new bone formation [22]. Another study investigated the influence of the pore shape on mechanical properties and showed that the cubic scaffold was conductive to osseointegration and tissue integration [23].

Given that the surface of severe acetabular bone defects was not entirely cancellous bone, the defect surface of many revision THA patients would experience partial corticalization due to long-term wear. Therefore, the pore parameters in the current study were a compromise between the mechanical and biological considerations, i.e., cubic-shaped lattice structure, with a pore size of 400 *μ*m, a strut size of 200 *μ*m, and a porosity of 60%. After printing by direct metal laser sintering (DMLS), the porous Ti6Al4V augments, with a total porosity of 55.48 ± 0.61% and a pore size of 319.23 ± 25.05 *μ*m, were used in this study. And the compressive strength and elastic modulus of the porous Ti6Al4V augments were 231.10 ± 11.77 MPa and 5.35 ± 0.23 GPa, respectively. These porous parameters of the 3D printed Ti6Al4V augments were favorable for bone tissue integration, and their mechanical properties also fit those of the human cortical bone in terms of elasticity.

The ultimate goal of bone defect repair by porous prostheses is to attain osseointegration between implant and human bone and long-term biological fixation [13, 24, 25]. Thomsen et al. revealed that the bone-implant contact, 6 weeks after surgery, was 29-41% in the femoral and tibial bone defect of rabbits [24]. A long-term sheep experiment by Palmquist et al. demonstrated that the bone-implant contact, 26 weeks after implantation, was up to 57% [25]. Ponader et al. examined the direct contact between the bone and implant surfaces to assess the ingrowth of osseous tissue inside the porous structure (a porosity of 61.3% and a pore size of 450 *μ*m) and found that the volume of newly formed bone tissue inside implants 14 days, 30 days, and 60 days after implantation was roughly 14.44%, 29.46%, and 46.31%, respectively [13]. The percentage bone volume of new bone in our study 12 weeks after surgery was 22.30 ± 4.51%, and the bone mineral apposition rate was 3.77 ± 0.93 *μ*m/d, which was consistent with previously reported findings [13, 24, 25].

The ultimate shear strength and the minimum load that separates bone from the augment are effective indicators of stability of the implanted augment, since they objectively reflect the adhesive strength between the augment and the newly formed bone tissues. The ultimate shear strength in our study immediately and 12 weeks after surgery was 929.46 ± 295.99 N and 1521.93 ± 98.38 N (*p* = 0.0302), respectively. The body weight of the miniswine in our study was 25-30 kg, while the mean shear strength immediately after surgery was 929.46 N (approximately 90 kg body weight), which was three times the body weight of a miniswine. Consequently, the immediate stability between the bone and the augment sufficed to support the daily activity of miniswine. As to the volume of newly formed bone inside the porous augment, the shear strength increased to 1521.93 N 12 weeks after the operation.

These results suggested that the 3D printed porous Ti6Al4V augments fabricated in this study had good bone tissue biocompatibility and biomechanical properties. In addition, our previous study on the finite element analysis also indicated that the periacetabular bone strength was adequate to support the patients' single-legged standing immediately after surgery [17]. Moreover, the postoperative three-dimensional reconstruction of CT data showed that the porous augment anatomically matched well with the acetabular bone defect.

This study had several limitations. First, only one type of acetabular bone defect (Paprosky IIB) was created in the current animal experiments. The Paprosky IIB type bone defect only represents the injury of the dome region of the acetabulum with the biggest shear strength, when compared to other types of acetabular bone defects. Second, the uncontrolled nature of the study prevented us from proving the advantages of the 3D printed porous Ti6Al4V augments over other alternatives. However, the positive results in both the animal models made us believe that the 3D printed porous Ti6Al4V augment is an effective choice for managing severe acetabular bone defects.

In summary, the 3D printed porous Ti6Al4V augment presented good bone tissue biocompatibility and biomechanical properties in our animal model. These augments anatomically well matched with the defect bone. Therefore, the 3D printed porous Ti6Al4V augment possesses great potential as an alternative for individualized treatment of severe acetabular bone defects.

## Figures and Tables

**Figure 1:** Representative pictures showing the establishment of the acetabular bone defect model and implantation of the 3D printed porous Ti6Al4V augment into miniswine. (a) The size of the acetabular bone defect was determined by a ruler. (b) The anterosuperior wall of the acetabulum was exposed clearly. (c) The bone defect model was completely created (the yellow triangle). (d) The size of the osteotomized bone was measured. (e) The 3D printed porous Ti6Al4V augment was temporarily fixed by two K-wires. (f) Two screws were inserted into the augment screw holes.

**Figure 2:** The graphical illustration of the design of the 3D printed porous Ti6Al4V augment and the micro-CT imaging of the acetabulum along with the augment taken from miniswine 3 months after implantation. (a) The thickness of the porous Ti6Al4V coating was 1 mm, and the rest of the augment was solid Ti6Al4V. (b) The designed length of screws was 16-20 mm. (c) The designed direction of screws. (d) The final design of the 3D printed porous Ti6Al4V augment fixed on the acetabulum. (e) The micro-CT imaging showing bone formation within the porous augments, and the specimen was taken 12 weeks after surgery (the inset in the upper-right corner). (f) The enlarged photo of the 3D printed porous Ti6Al4V augment.

**Figure 3:** The graphical illustration of the calculation of matching degree with the three-dimensional reconstruction of the augment as shown by CT scans, and the values of matching degree in individual swine. (a) Postoperative CT scan identified the screw direction. (b) The overlapping ranges of designed and implanted augments and screws. (c, d) The implanted augment matched with the defect bone surface (blue, implanted augment; golden yellow, designed augment). (e) The matching degrees of implanted augments in individual swine, with the mean ± SD value being 91.40 ± 3.01% (*n* = 9).

**Figure 4:** Representative pictures showing the platform for the push-out test and the results of the push-out test in 3 swine. (a) The pictures of the mechanical testing platform for the push-out test. (b) The ultimate shear strength immediately (0 weeks) and 12 weeks after surgery. *p* < 0.05 (*n* = 3).

**Figure 5:** Histological and histomorphometric analyses of the implanted augment 12 weeks after implantation. (a) The newly formed bone was determined by the distance between the two fluorochrome labels (tetracycline and calcein green bands) using an epifluorescent microscope. (b) The amount of new bone and bone ingrowth to the interior of the pores was calculated using image processing software, presented as a percentage of the total bone-implant interface area. (c) Bone mineral apposition rate (MAR) was 3.77 ± 0.93 *μ*m/d (*n* = 3; the numbers indicate the values in three individual swine). (d) Percentage bone volume of new bone (Tb/T) 12 weeks after surgery was 22.30 ± 4.51% (*n* = 3; the numbers indicate the values in three individual swine).

## Data Availability

The datasets used and/or analyzed during the current study are available from the corresponding authors on reasonable request.

## References

[1] Kurtz S., Ong K., Lau E., Mowat F., Halpern M. (2007). Projections of primary and revision hip and knee arthroplasty in the United States from 2005 to 2030. *The Journal of Bone and Joint Surgery-American Volume*.

[2] Shon W. Y., Santhanam S. S., Choi J. W. (2016). Acetabular reconstruction in total hip arthroplasty. *Hip & Pelvis*.

[3] Cuckler J. M. (2002). Management strategies for acetabular defects in revision total hip arthroplasty. *The Journal of Arthroplasty*.

[4] Fernandez-Fairen M., Murcia A., Blanco A., Merono A., Murcia A., Ballester J. (2010). Revision of failed total hip arthroplasty acetabular cups to porous tantalum components: a 5-year follow-up study. *The Journal of Arthroplasty*.

[5] Sporer S. M., Paprosky W. G. (2006). The use of a trabecular metal acetabular component and trabecular metal augment for severe acetabular defects. *The Journal of Arthroplasty*.

[6] Whitehouse M. R., Masri B. A., Duncan C. P., Garbuz D. S. (2015). Continued good results with modular trabecular metal augments for acetabular defects in hip arthroplasty at 7 to 11 years. *Clinical Orthopaedics and Related Research*.

[7] Swaminathan V., Gilbert J. L. (2012). Fretting corrosion of CoCrMo and Ti6Al4V interfaces. *Biomaterials*.

[8] Li J., Li W., Li Z. (2019). In vitroandin vivoevaluations of the fully porous Ti6Al4V acetabular cups fabricated by a sintering technique. *RSC Advances*.

[9] Zhang B., Pei X., Zhou C. (2018). The biomimetic design and 3D printing of customized mechanical properties porous Ti6Al4V scaffold for load-bearing bone reconstruction. *Materials & Design*.

[10] Kujala S., Ryhänen J., Danilov A., Tuukkanen J. (2003). Effect of porosity on the osteointegration and bone ingrowth of a weight-bearing nickel–titanium bone graft substitute. *Biomaterials*.

[11] Wang J., Yang M., Zhu Y., Wang L., Tomsia A. P., Mao C. (2014). Phage nanofibers induce vascularized osteogenesis in 3D printed bone scaffolds. *Advanced Materials*.

[12] Kalantari S. M., Arabi H., Mirdamadi S., Mirsalehi S. A. (2015). Biocompatibility and compressive properties of Ti-6Al-4V scaffolds having Mg element. *Journal of the Mechanical Behavior of Biomedical Materials*.

[13] Ponader S., Von Wilmowsky C., Widenmayer M. (2010). In vivo performance of selective electron beam-melted Ti-6Al-4V structures. *Journal of Biomedical Materials Research Part A*.

[14] Ramakrishnaiah R., al kheraif A. A., Mohammad A. (2017). Preliminary fabrication and characterization of electron beam melted Ti-6Al-4V customized dental implant. *Saudi Journal of Biological Sciences*.

[15] Honigmann P., Sharma N., Okolo B., Popp U., Msallem B., Thieringer F. M. (2018). Patient-specific surgical implants made of 3D printed PEEK: material, technology, and scope of surgical application. *BioMed Research International*.

[16] Lal H., Patralekh M. K. (2018). 3D printing and its applications in orthopaedic trauma: a technological marvel. *Journal of Clinical Orthopaedics and Trauma*.

[17] Fu J., Ni M., Chen J. (2018). Reconstruction of severe acetabular bone defect with 3D printed Ti6Al4V augment: a finite element study. *BioMed Research International*.

[18] Smith A. C., Swindle M. M. (2006). Preparation of swine for the laboratory. *ILAR Journal*.

[19] Paprosky W. G., Perona P. G., Lawrence J. M. (1994). Acetabular defect classification and surgical reconstruction in revision arthroplasty: a 6-year follow-up evaluation. *The Journal of Arthroplasty*.

[20] Heinl P., Muller L., Korner C., Singer R. F., Muller F. A. (2008). Cellular Ti–6Al–4V structures with interconnected macro porosity for bone implants fabricated by selective electron beam melting. *Acta Biomaterialia*.

[21] Srivas P. K., Kapat K., Dadhich P. (2017). Osseointegration assessment of extrusion printed Ti6Al4V scaffold towards accelerated skeletal defect healing via tissue in-growth. *Bioprinting*.

[22] Wieding J., Wolf A., Bader R. (2014). Numerical optimization of open-porous bone scaffold structures to match the elastic properties of human cortical bone. *Journal of the Mechanical Behavior of Biomedical Materials*.

[23] Schumacher M., Deisinger U., Detsch R., Ziegler G. (2010). Indirect rapid prototyping of biphasic calcium phosphate scaffolds as bone substitutes: influence of phase composition, macroporosity and pore geometry on mechanical properties. *Journal of Materials Science: Materials in Medicine*.

[24] Thomsen P., Malmström J., Emanuelsson L., Rene M., Snis A. (2009). Electron beam-melted, free-form-fabricated titanium alloy implants: material surface characterization and early bone response in rabbits. *Journal of Biomedical Materials Research Part B: Applied Biomaterials*.

[25] Palmquist A., Snis A., Emanuelsson L., Browne M., Thomsen P. (2013). Long-term biocompatibility and osseointegration of electron beam melted, free-form-fabricated solid and porous titanium alloy: experimental studies in sheep. *Journal of Biomaterials Applications*.

